# Analysis of Clinical Characteristics of Hepatitis B and Alcohol-Related Liver Cancer

**DOI:** 10.1155/2021/9752534

**Published:** 2021-11-18

**Authors:** Yuefei Pan, Guiliang Han

**Affiliations:** ^1^Department of Disease Control and Prevention, The 81st Group Army Hospital of the PLA Army, Zhangjiakou 075000, China; ^2^Hebei Key Laboratory of Cancer Radiotherapy and Chemotherapy, Department of Medical Oncology, Affiliated Hospital of Hebei University, Baoding 071000, China

## Abstract

In order to analyze the clinical characteristics of hepatitis B and alcohol-related liver cancer, this paper combines the investigation and analysis methods to analyze the clinical characteristics of hepatitis B and alcohol-related liver cancer, studies them in combination with the actual situation, and studies multiple parameters with statistical methods. Different causes of liver cancer have different pathogenic mechanisms, which may make the clinical characteristics of liver cancer different. This study mainly explores the difference in clinical characteristics between hepatitis B-related hepatocellular carcinoma and alcohol-related hepatocellular carcinoma. Through comparative analysis and analysis of the clinical characteristics of hepatitis B and alcohol-related liver cancer, the study found that hepatitis B and alcohol-related liver cancer have obvious differences in their impact mechanisms. Therefore, targeted prevention and diagnosis and treatment measures can be put forward on this basis to provide a theoretical reference for subsequent clinical treatment analysis of liver cancer.

## 1. Introduction

Primary carcinoma of the liver (PLC) is a frequent malignant tumor in my nation and across the globe that develops from a mixture of liver cells, intrahepatic bile duct epithelial cells, or hepatocytes and intrahepatic bile duct epithelial cells. PLC patients are increasing at a pace of 626,000 per year worldwide, and PLC deaths account for 51% of all deaths in my country [1]. PLC has a high mortality rate, and it ranks second among malignant tumors in terms of fatality rate in my country [2]. In my country, persistent HBV infection is responsible for about 90% of PLC cases [3]. PLC has placed a significant financial load on our nation and has put our people's life and health in jeopardy. The origin and pathophysiology of PLC are not completely known in the globe because of existing medical limitations. Chronic viral infection of the liver, cirrhosis, frequent eating of aflatoxins-contaminated food, long-term drinking of algae-toxin-contaminated drinking water, genetic variables associated with liver cancer, alcohol, toxic chemicals, and liver fluke infections are all possible causes. Chronic persistent infection of HBV is the main pathogenic factor of PLC in our country, but the most common pathogenic factor in western countries is alcohol. The pathogenesis of PLC may be as follows. One is the activation of proto-oncogenes and mutations of tumor suppressor genes. On the other hand, the latest HBV pathogenesis shows that HBV integrates with human chromosomes in liver cells, and HBV's X protein as an enhancer can transactivate cancer genes such as c-jun and c-myc to promote integrated liver cell transformation. China's PLC cases account for more than half of the global cases, and they are prone to relapse after surgery, high mortality, and short survival. PLC has seriously affected the lives and health of patients and has attracted great attention from people all over the world, and a series of studies have been carried out.

Chronic hepatitis B infection is the leading cause of liver cancer. Hepatitis B virus is responsible for 70 percent to 80 percent of liver malignancies. The annual incidence of liver cancer in noncirrhotic HBV-infected people is 0.5-1.0 percent, while the annual incidence of liver cancer in HBV-infected patients with cirrhosis is 3 percent -6 percent. In the literature, the clinical signs of HBV-HCC and HCV-HCC have been shown to be significantly different. Between the ages of 50 and 59, HBV-HCC occurs, while HCV-related HCC develops gradually until the age of 70. At the time of diagnosis, HBV-HCC is also identified. HCV-HCC multiple tumors are more frequent, as are large-volume tumors and portal vein involvement. Except for advanced tumors, there is no difference in survival prognosis between the two. Gender, Child-Pugh classification of liver function, AJCC/UICC staging, and treatment methods are independent risk factors associated with the survival of HBV and HCV-related HCC. Domestic studies have shown that tumor size, AFP level, tumor BCLC staging, and serum iron level are independent risk factors that affect the prognosis of hepatitis B virus-related liver cancer. Patients in the HBV-HCC group have a younger age of onset and poor liver function. Compared with nonviral-related liver cancer, HBV-HCC has a worse prognosis. The overall survival rates of 1, 3, and 5 years are 76.7%, 52.4%, and 52.4%, respectively. 42.5% are with a median survival time of 40 months. The low survival rate of HBV-HCC is related to its high recurrence rate. The recurrence rate is as high as 50%-70% in 5 years after radical surgery. In addition to AFP, tumor size, and other risk factors for recurrence, HBV-DNA load is also closely related to it, and studies have shown that HBV-DNA load is positively correlated with HBV-HCC mortality. As a result, antihepatitis B virus therapy that reduces HBV-DNA is critical in lowering liver cancer mortality.

The main causes of liver cancer are HBV, HCV infection, and alcoholic liver disease. With changes in diet and lifestyle, the incidence of NAFLD-related liver cancer is on the rise, although nonalcoholic fatty liver has become more and more primary liver cancer. Important risk factors but viral hepatitis B and alcohol abuse are still the main pathogenic factors in China. There are few reports on the clinical characteristics and prognosis of ALC-HCC and HBV-HCC in domestic and foreign literature. At present, it is not known what the clinical characteristics and prognosis of ALC-HCC and HBV-HCC are different, so the comparison of primary liver cancer caused by two different etiologies is particularly important. This research compared the numerous clinical variables of the two groups of liver cancer patients with distinct etiologies in more depth in order to better understand the two and offer clinical evidence for their prevention and therapy.

## 2. Related Work

Hepatitis B virus (HBV) is a DNA virus and belongs to the family of hepatotropic DNA viruses. The full length of the genome is about 3.2 kb. It is a partially double-stranded circular DNA molecule and is currently the smallest DNA virus known to infect humans [4]. The HBV genome is small, only 3.2 kb in size, but it contains many promoters, enhancers, and 4 main open reading frames (S, C, P, X). HBsAg, as a marker of HBV infection in the serum, is produced by the S gene. HBcAg is produced after the C gene is encoded. The antibody corresponding to HBcAg is HBcAb, which is the earliest antibody after HBV infection. The P protein is made by the P gene. It is a straightforward protein with many functional parts. The X protein is encoded by the X gene, which has transcriptional activation activity [5]. Chronic HBV infection is the leading cause of liver cancer. After HBV infects liver cells, its DNA sequence may be integrated with the host DNA sequence, resulting in proto-oncogene activation or tumor suppressor gene silencing. This is the catalyst for hepatocellular carcinogenesis and the molecular foundation for HCC development. Telomerase reverse transcriptase (TERT) was the first to identify the HBV integrated insert gene, according to the literature [6]. After activation, HBV DNA integration near TERT causes the TERT gene to become overexpressed, promoting tumor cell transformation and the development of liver cancer. In addition, common HBV DNA integration insert genes include granulocyte/lymphoid or mixed-lineage leukemia 4 (myeloid/lymphoid or mixed-lineage leukemia 4, and MLL4) and cyclin E1 (cyclin E1 and CCNE1). After HBV DNA is integrated into the host DNA, it also affects the stability of the host gene. The literature [7] found that HBV DNA integration caused mutations in chromosome regulatory genes, causing chromosomes to appear aberrations, which are structurally manifested as deletions, amplifications, and ectopic copy number variations. X gene can be incorporated into human cells more readily and stably than the other three genes, according to studies, and maintain transcriptional activity. By activating and regulating tumor-related genes, preventing tumor cell death, and altering cytogenetic expression, the HBx protein may promote the development of HCC. In liver cells, a variety of kinases and signal transduction pathways are affected by HBX protein. For example, the activation of extracellular signal-regulated kinase (ERK), NF-*κ*B, JAK-STAT signaling pathway, Wnt/*β*-catenin pathway, etc. can upregulate the expression of tumor-related factors, thereby promoting cell growth and transformation, and ultimately leading to the formation of HCC [8]. HBx may affect the function of certain tumor suppressor genes and their proteins and promote the occurrence of HCC. The HBX protein binds to the tumor suppressor gene P53, the protein complex formed by it can inhibit the transcription of P53, and the activation of genes such as p21 and fas in the downstream apoptotic pathway can also be inhibited [9]. According to the literature [10], HBx may directly control the anchoring region of the P53 target gene, causing it to change and disrupting P53's normal function. Furthermore, HBX may regulate DNA methyltransferase transcription, resulting in hypermethylation of the promoter DNA region of tumor formation-related genes with CpG islands, inactivation of tumor suppressor genes, and increased HCC risk. DNA methylation can occur simultaneously with histone modifications such as acetylation. HBX acts on histone deacetylases to stimulate epigenetic modifications of tumor-related genes and induce the occurrence of HCC [11]. HBx can also promote the occurrence of HCC by changing the expression of certain microRNAs. HBx can upregulate the expression of miRNAs that is conducive to tumor formation, such as miR-602 and miR148a. Moreover, it can also downregulate the expression of miRNAs that inhibit tumor formation, such as miR-122 and miR-373 [12].

With the continuous increase in alcohol consumption, chronic alcohol abuse has become a major risk factor for the occurrence of HCC, but previous studies have not yet fully clarified its specific pathogenic mechanism. It is currently believed that chronic alcohol abuse may lead to alcoholic liver disease through a variety of ways, and then alcoholic cirrhosis develops and eventually progresses to liver cancer. After drinking, 80% of ethanol is quickly absorbed. In liver cells, it is metabolized into acetaldehyde under the action of alcohol dehydrogenase (ADH) and cytochrome P450 2E1 (CYP2E1). Acetaldehyde forms a complex with DNA to initiate replication. Error; acetaldehyde forms a complex with protein, which changes the structure and function of protein [13]. Acetaldehyde can also stimulate the synthesis of collagen in hepatic stellate cells to promote the occurrence of liver cirrhosis and eventually develop into HCC [14]. Chronic consumption of alcohol can double CYP2E1. Under the induction of CYP2E1, reactive oxygen species (ROS), lipid peroxidation, malondialdehyde (MDA), and 4-hydroxynonenal (4-HNE) levels will also increase. These products work together to form a DNA polymer with mutagenic potential [15]. In addition, alcohol may also cause liver cancer through DNA methylation, immune mechanism, inflammation, and other ways. Under the induction of alcohol, the methyl donor S-adenosylmethionine (SAMe) level decreases and the S-adenosyl homocysteine (SAH) level increases, which reduces SAMe/SAH and promotes carcinogenesis [16]. Literature [17] shows that Toll-like receptor 4 (TLR4) is involved in mediating the carcinogenic effects of alcohol and NS5A. Severe alcohol intake increases the permeability of the intestinal mucosa to lipopolysaccharide (LPS), thereby increasing the level of LPS in the liver. LPS binds to the CD14 and TLR4 complex of Kupffercells (KC), resulting in proinflammatory cytokines The release of tumor necrosis factor-*α* (TNF-*α*) and transforming growth factor b (TGF-b), etc., caused liver cell damage. Alcohol abuse can directly induce the occurrence of liver cancer. However, the risk of cancer caused by alcohol alone is relatively small. If HBV or HCV infection is combined with alcohol abuse, the risk of liver cancer will increase significantly [18].

## 3. Research Method

This article collects clinical data of patients with hepatitis B-related liver cancer and alcohol-related liver cancer diagnosed for the first time from January 2018 to June 2021. According to the inclusion criteria and exclusion criteria, they are finally included in this study.

1. *General Information*. Gender, age, history of antiviral treatment, family history of liver cancer, history of drinking, history of liver fluke infection, history of liver cirrhosis, clinical symptoms (abdominal pain, diarrhea, bloating, and weight loss), and physical signs (jaundice, ascites, and hepatomegaly)
2. *Auxiliary Examination and Clinical Data*. Clinicopathological classification (massive, nodular, and diffuse), histopathological classification (hepatocyte, cholangiocytic, and mixed), hepatitis B surface antigen (HBsAg), hepatitis B surface antibody (HBsAb), hepatitis B e antigen (HBeAg), hepatitis B e antibody (HBeAb), hepatitis B core antibody (HBcAb), TBIL, ALT, AST, ALB, AFP, PT, Child-Pugh score, and HBV DNA

The age of the two groups of patients, family history of liver cancer, history of drinking, history of liver fluke infection, history of liver cirrhosis, symptoms (abdominal pain, diarrhea, bloating, and weight loss), physical signs (jaundice, ascites, and hepatomegaly), clinicopathological classification (massive, nodular, and diffuse), clinicopathological classification (massive, nodular, and diffuse), histopathological classification (massive, nodular, and diffuse), histopathological classification (hepatocyte, cholangiocytic, and mixed), TBIL, ALT, AST, ALB, AFP, PT, and Child-Pugh score.

The collected case data are processed and analyzed using Excel tables, and statistical analysis is performed using SPSS 17.0 statistical software. Measurement data are represented as mean standard deviation (*x* *s*), and the two groups are compared using an independent sample *t* test, with *P*0.05 indicating that the difference is statistically significant. The comparison of count data is performed by *χ*^2^ test, and *P* ≤ 0.05 is considered statistically significant.

## 4. Result

Among patients with hepatitis B-related liver cancer, 86.47% are males and 13.53% are females. For alcohol-related liver cancer patients, 100% are males and 0.0% are females. The results are shown in Figures 1 and 2.

The age distribution of hepatitis B-related liver cancer and the age distribution of alcohol-related liver cancer are shown in Figures 3 and 4, respectively.

The personal history of this study includes a history of drinking, a history of liver fluke infection, and a history of liver cirrhosis. The differences between the two groups of data were statistically significant (both *P* values < 0.05). The results are shown in Table 1 and Figure 5.

The comparison results of the clinical manifestations of the two groups of patients at the first visit are shown in Table 2 and Figure 6.

In the comparison of the clinicopathological classification of liver cancer (massive, nodular, and diffuse) between the two groups of liver cancer patients, the difference was not statistically significant (*P* > 0.05), as shown in Table 3 and Figure 7.

In the comparison of the histopathological classification of liver cancer (hepatocellular type, cholangiocytic type, and mixed type) between the two groups of liver cancer patients, the difference was not statistically significant (*P* > 0.05), as shown in Table 4 and Figure 8.

## 5. Analysis and Discussion

The proportion of male patients with PLC reported in this study is higher than that generally reported. There is a statistically significant difference between hepatitis B-related liver cancer and alcohol-related liver cancer in the comparison of drinking history (*P* < 0.05). The results suggest that the proportion of alcohol-related liver cancer patients' drinking history is much higher than that of hepatitis B-related liver cancer, and PLC is closely related to patients' long-term drinking. Hepatitis B and alcohol-related liver cancer mainly occur in male patients, and the reasons may be as follows. (1) In terms of chronic persistent HBV infection, men have a higher degree of HBV replication than women. Estrogen may block hepatitis B virus X protein (HBx) and estrogen receptor variants missing exon 5, preventing hepatoma cell estrogen receptor signal transduction, hepatitis B virus replication, and PLC. Androgens can induce the replication of HBV and promote the occurrence of PLC. (2) It may be related to the drinking of male patients. Drinking is a risk factor for PLC, and drinking increases the risk of PLC. (3) Alcohol can aggravate the chronic inflammation of the liver, accelerate the malignant transformation of the liver, and lead to the occurrence of PLC. Alcohol and HBV can synergistically promote the occurrence of PLC. Alcohol increases the oxygen stress of the liver, aggravates the liver damage associated with HBV infection, and reduces the liver's detoxification and excretion capacity. The reason why the alcohol-related liver cancers in this study are all male patients may be related to the higher drinking rate of male patients. However, the safety threshold of women for alcohol is significantly lower than that of men. Therefore, women who have a history of hepatitis B and drinking history should also be highly concerned.

Around 25% of individuals infected with HBV before the age of 6 may develop PLC later in life, while the majority of HBV infections in my country are caused by infections in babies and children. The incidence of hepatitis B-related liver cancer is positively correlated with the course of HBV infection. The earlier the patient is infected with HBV, the earlier it is likely to progress to liver cirrhosis and PLC. Therefore, for young patients with a long history of HBV infection, follow-up and early screening should be strengthened.

Research reports show that more than 80% of the causes of PLC are the development of hepatitis and liver cirrhosis patients. However, the incidence of cirrhosis-related hepatitis B-related liver cancer in this research is considerably lower than previously published statistics. Therefore, patients with chronic hepatitis B without cirrhosis should also be alert to the occurrence of PLC to prevent missed diagnosis and delay in treatment. In this study, the rate of patients with hepatitis B-related liver cancer and cirrhosis was significantly lower than the reported data. The reasons may be as follows: clinical diagnosis is not difficult to diagnose decompensated cirrhosis through the patient's medical history, symptoms and signs, laboratory examinations, and auxiliary examinations. The clinical diagnosis of compensated cirrhosis is often difficult. Compensated cirrhosis often requires liver biopsy to confirm the diagnosis. Because liver biopsy is a traumatic invasive examination and is often not accepted by patients, it is easy to lead to missed diagnosis of compensated cirrhosis. The direct cause of PLC after HBV infection is not yet clear, and the pathogenesis may be as follows. (1) Chronic and persistent HBV infections activate the HBx gene, which further leads to the activation of cancer genes and the inactivation of tumor suppressor genes. (2) Chronic and persistent HBV infections have caused mutations in P53, P16, and pre-C genes. Although chronic and persistent HBV infections does not have the basis of liver cirrhosis, and it can still directly evolve into PLC.

Therefore, patients with hepatitis B who are clinically diagnosed with no cirrhosis should also pay attention to regular investigations for the presence of PLC to prevent missed diagnosis. Chronic persistent infection of HBV is the main pathogenic factor of PLC, and the most common pathogenic factor in western countries is alcohol. The history of HBV infection is the most important cause of hepatitis B cirrhosis and PLC. In my nation, the HBV infection rate of PLC may approach 90%, suggesting that PLC and HBV infection are linked. Patients with hepatitis B-related liver cancer and cirrhosis are more likely to suffer perioperative liver failure and mortality, according to the findings of a comparative study. As a result, patients with hepatitis B-associated liver cancer and cirrhosis should focus more on assessing surgical risks and preparing for relevant procedures prior to surgery.

There was no statistical difference in the cause of liver fluke infection between the two groups of patients with liver cancer. Liver fluke infection is closely related to the onset of PLC. Liver fluke infection is Clonorchis sinensis infection, and the history of liver fluke infection is one of the causes of PLC. Patients infected with liver flukes were mainly due to eating foods containing live metacercariae of liver flukes, such as immature freshwater fish and shrimp, raw fish, and cross-contamination between raw and cooked foods. Liver flukes are mainly parasitic in the intrahepatic bile ducts after infection, which can cause abdominal pain, bloating, diarrhea, indigestion, and other symptoms. However, the milder can also have no symptoms. The mechanism of liver fluke infection leading to PLC is not yet fully understood. The reason may be as follows. After liver fluke infection, it damages bile duct endothelial cells, and repeated stimulation causes continuous inflammation, cholestasis, and bacterial infection of bile duct endothelial cells, thereby producing a series of inflammatory substances, which further stimulate the formation of tumor cells. If the patient is infected with HBV, liver fluke infection can further aggravate liver cell damage. With time, it can progress to liver cirrhosis and PLC. Therefore, clinical attention should be paid to screening liver disease for liver fluke infection. A standardised deworming therapy can eliminate all liver fluke infections, minimising liver cell damage, increasing liver function, and decreasing the risk of PLC.

The *P* value for the comparison of the family history of liver cancer between the two groups was less than 0.05, so the difference was statistically significant. The results of this study suggest that the proportion of patients with hepatitis B-related liver cancer with a family history of liver cancer is significantly higher than the proportion of patients with alcohol-related liver cancer with a family history of liver cancer. Family history of liver cancer refers to the incidence of liver cancer in the patient's family, and HBV infection combined with family history of liver cancer is an important risk factor leading to the onset of PLC. The risk of PLC in HBsAg-positive patients with a family history of hepatitis B liver cancer is significantly higher than that of HBsAg-positive patients without a family history of liver cancer. As a result, HBsAg-positive individuals with a family history of liver cancer should have an AFP, abdominal ultrasound, upper abdominal CT, upper abdominal MRI, and other tests done at least once every 6 months to screen for PLC.

The onset of PLC is insidious. When the patient has clinical manifestations such as abdominal pain, bloating, diarrhea, ascites, jaundice, and weight loss, the disease often enters the middle and late stages. The symptoms of PLC abdominal pain are mostly persistent dull pain and distending pain, which are caused by the liver capsule being stretched due to the rapid growth of liver cancer tissue. If the liver cancer tissue grows slowly, there may be no symptoms of abdominal pain. When the cancer nodules in the liver rupture and hemorrhage, it can cause sudden abdominal pain and acute abdomen and even cause shock and death. The symptoms of abdominal distension are mostly related to gastrointestinal dysfunction, indigestion, and flatulence. When decompensated liver cirrhosis causes a large amount of ascites, the symptoms of abdominal distension are often obvious. Viral hepatitis, liver cirrhosis, primary peritonitis, chronic gastritis, peptic ulcer, cholecystitis, etc. can also cause abdominal pain and bloating. Therefore, attention should be paid to identify the cause of abdominal pain and bloating to prevent missed diagnosis of PLC, thereby delaying the patient's treatment. Patients experiencing stomach discomfort and bloating, particularly those with a history of chronic HBV infection and a long-term drinking history, should be screened for PLC more often.

The *P* value of the clinical classification of liver cancer between the two groups is greater than 0.005, so the difference is not statistically significant. The most common clinical classification of PLC is the massive type. The massive type has a diameter of more than 5 cm, and the one greater than 10 cm is considered to be a massive type. Massive liver cancer is prone to liquefaction, necrosis, and bleeding due to the formation of a pseudocapsule. It is often accompanied by rupture and bleeding of cancer nodules, which can lead to acute abdominal pain and acute abdomen, and even shock and death. The most common clinical classification is the massive type, and the clinicians should pay great attention to the complications of massive liver cancer that may cause liver cancer rupture and bleeding. The main clinical classification of PLC is block type. Moreover, the larger the diameter of the liver cancer tumor, the worse the prognosis and the shorter the survival period.

## 6. Conclusion

Hepatitis B-related liver cancer has a high incidence age group of 40-59 years old, while alcohol-related liver cancer has a high incidence age group of 50-69 years old. Hepatitis B-related liver cancer develops at a younger age than alcohol-related liver cancer, and the age of onset is on the rise. PLC is caused by a combination of chronic HBV infection and alcohol use, which may exacerbate liver damage and lead to the development of PLC. Abdominal pain and bloating are the first significant clinical signs of PLC, although abdominal discomfort and bloating may also be caused by chronic gastritis, peptic ulcer, hepatitis, liver cirrhosis, cholecystitis, and other conditions. To avoid missing a diagnosis, it is important to pay attention to the reasons of stomach discomfort and bloating. The “small three positives” infection pattern is dominant in hepatitis B-related liver cancer, although the negative rate of HBV DNA in patients with “small three positives” is greater. It is possible that this is because “small three positive” people have viral mutations and have been infected for extended periods of time, and long-term chronic HBV infection is more likely to produce PLC. Furthermore, patients with the “little three positives” have a high HBV DNA negative rate, prompting physicians to disregard antiviral therapy.

## Figures and Tables

**Figure 1:** Gender distribution of hepatitis B-related liver cancer.

**Figure 2:** Gender distribution of alcohol-related liver cancer.

**Figure 3:** Age distribution of hepatitis B-related liver cancer.

**Figure 4:** Age distribution of alcohol-related liver cancer.

**Figure 5:** Comparison of personal history and family history of liver cancer between the two groups.

**Figure 6:** Statistical diagram of clinical manifestations.

**Figure 7:** Statistical diagram of clinical classification of liver cancer.

**Figure 8:** Statistical diagram of comparison of histopathological classification of two groups of patients with liver cancer.

**Table 1:** Comparison of personal history and family history of liver cancer between the two groups.

Compare items	Hepatitis B-related liver cancer	Alcohol-related liver cancer	*P*
Drinking history (%)	24.8	100	0
History of liver fluke infection (%)	12.8	14.5	0.74
History of liver cirrhosis (%)	44.9	53.8	0.264
Family history (%)	35.8	5.1	0

**Table 2:** Comparison table of clinical manifestations of the two groups of patients.

	Stomach ache	Diarrhea	Bloating	Thin	Jaundice	Ascites	Hepatomegaly
Hepatitis B-related liver cancer	60.62%	13.62%	51.36%	28.43%	15.17%	24.44%	29.56%
Hepatitis B-related liver cancer	49.59%	10.61%	53.13%	33.63%	17.68%	24.85%	31.92%
*χ* ^2^	2.823	4.242	0.031	0.612	0.217	0.001	0.097
*P*	0.096	0.522	0.869	0.440	0.649	0.989	0.765

**Table 3:** Comparison of clinical classification of liver cancer between the two groups.

	Block type	Nodular	Diffuse
Hepatitis B-related liver cancer	60.80%	30.7%	8.50%
Hepatitis B-related liver cancer	56.40%	38.50%	5.10%

**Table 4:** Comparison results of histopathological classification of two groups of patients with liver cancer.

	Hepatocyte type	Cholangiocytic type	Hybrid
Hepatitis B-related liver cancer	84.50%	11.80%	3.70%
Hepatitis B-related liver cancer	80%	18%	2%

## Data Availability

The data used to support the findings of this study are included within the article.
